This article has been retracted.

# Sole and combined effect of foliar zinc and arbuscular mycorrhizae inoculation on basmati rice growth, productivity and grains nutrient

**DOI:** 10.1371/journal.pone.0266248

**Published:** 2022-04-29

**Authors:** Hassan Mehmood, Muhammad Arif Ali, Saddam Hussain, Khurram Shehzad Baig, Haider Sultan, Syed Atif Hasan Naqvi, Muhammad Nadeem Shahid, Shamsher Ali, Eman A. Alhomaidi, Rahul Datta

**Affiliations:** 1 Department of Soil Science, Faculty of Agricultural Sciences and Technology, Bahauddin Zakariya University, Multan, Punjab, Pakistan; 2 Department of Agronomy, University of Agriculture, Faisalabad, Punjab, Pakistan; 3 Soil & Water Testing Laboratory, Muzaffargarh, Punjab, Pakistan; 4 Hainan Key Laboratory for Sustainable Utilization of Tropical Bioresource, College of Tropical Crops, Hainan University, Haikou, China; 5 Department of Plant Pathology, Faculty of Agricultural Sciences and Technology, Bahauddin Zakariya University, Multan, Pakistan; 6 Department of Soil and Environmental Sciences, Amir Muhammad Khan Campus Mardan, The University of Agriculture Peshawar, Khyber Pakhtunkhwa, Pakistan; 7 Department of Biology College of Science, Princess Nourah Bint Abdulrahman University, Riyadh, Saudi Arabia; 8 Department of Geology and Pedology, Faculty of Forestry and Wood Technology, Mendel University in Brno, Brno, Czech Republic; The University of Haripur, PAKISTAN

## Abstract

Mismanagement in foliar fertilizer application at different crop stages decreases the productivity of the crop. Likewise, higher application of phosphorus (P) beyond recommended application rates not only decrease zinc (Zn) uptake in rice but also increase fertilizer use cost. Inoculation of arbuscular mycorrhizae (AMF) may optimize the uptake of P and improve crops production via organic secretions. That’s why the current study was conducted to examine the individual and coordinated effects of 0.5% Zn (0.5Zn) foliar spray (tillering (T) and/or panicle (P) initiation stage) and AMF application. Application of foliar 0.5Zn at tillering+panicle stage remained significantly better for significant enhancement in plant height, spike length, gas exchange attributes and total chlorophyll contents than control. A significant decrease in electrolyte leakage Also validated the effectiveness of treatment 0.5ZnT+P compared to control. Compared to control, the maximum increase in N (14.5 and 25.7%), P (42.1 and 33.3%), K (22.2 and 30.0%) and Zn (19.3 and 27.8%) accumulation was also found in 0.5ZnT+P, with and without AMF, respectively. In conclusion, 0.5ZnT+P with AMF is a better approach than sole application of Zn at tillering or panicle initiation stages. Nevertheless, more investigations are suggested at field level under variable climatic zones to confirm the effectiveness of 0.5ZnT+P with AMF for improvement in rice growth and production.

## Introduction

Poor availability of micronutrients is one of the major hurdles to the achievement of optimum crop productivity [1–4], because these are essential for plants due to the active role in the improvement of photosynthesis, cell membrane structure, nucleic acid and lipid metabolism, hormone activity, protein synthesis, gene expression and defense [5–7]. Nonetheless, high soil pH and poor organic contents in arid and semi-arid areas are major causes of less micronutrients bioavailability [8–10]. Among variable micronutrients, role of Zn is vital in plants growth [11–13]. Zinc is known to be involved in several metabolic as well as structural activities of plants including respiration, photosynthesis, and chlorophyll synthesis [14–16]. Furthermore, enzymes i.e., lyases, classes; oxido-reductases, ligases, isomerase, transferases and hydrolases also require sufficient concentration of Zn for their optimum activities [17]. However, more than 50% of agriculture soils are considered deficient in Zn bioavailability [18].

To overcome this issue, scientists suggest the application of Zn as fertilizer [14–16, 19]. The majority of macro and micronutrients fertilizers are applied in soil [17, 20, 21]. However, deteriorated physical and chemical conditions decrease the nutrients use efficiency (NUE) i.e., nitrogen (30–50%), phosphorus (15–20%) and micronutrients (<2%) [22]. On the other hand, supplementation of micronutrients as the foliar application can play an imperative role in the improvement of nutrient use efficiency [15, 23]. Most of the micronutrients which are applied as foliar, actively become part of plants due to quick absorption in tissue. This method also minimizes the leaching losses and precipitation of micronutrients which are key immobilizing processing in soil [24]. Although potential benefits are majorly associated with the foliar application of micronutrients, the selection of crop stage for foliar application is of prime importance. It is important to identify the potential yield describing the time period in the cultivated crop for the achievement of favorable post-reproductive development by foliar application of micronutrients [22].

The poor management of phosphate fertilizers in soils also decreases Zn availability to the plants. When phosphate fertilizers are applied in large amounts, they make complexes with Zn and decreases their uptake in the plants [25]. Inoculation of arbuscular mycorrhizae (AMF) is considered helpful in avoiding any disturbance in the balance uptake of phosphorus (P) [1, 26]. AMF significantly improve the root elongation, which increases the rhizosphere area where organic secretions regulate the balance uptake of P in plants [11]. Furthermore, improvement in soil characteristics due to improvement in the population of AMF in the soil also facilitate the improvement in growth and yield of crops [26].

Rice is considered an important food in human’s diet, as more than 50 million people consume it for their daily intake [27]. It has a significant amount of essential nutrients i.e., N, K, Zn, P, Ca, Fe and Na [28]. A 100 grams of rice grains is considered a source of lipid (~0.3–0.5 g), protein (~6.3–7.1 g), fiber (~0.2–0.5 g), carbohydrate (~77–78 g), riboflavin (~0.02–0.06 mg), thiamine (~0.02–0.11 mg), niacin (~1.3–2.4 mg) and vitamin E (~0.075–0.30 mg) [28]. That’s why the current experiment was planned with the aim to check the critical developmental stages of rice for foliar application of Zn in the presence and absence of AMF. The study is covering the knowledge gap of the best developmental stage among panicle and tillering of rice for application of Zn with and without AMF inoculation situation. It is hypothesized that application of Zn at panicle and tillering stages in split may be a better approach than sole application at panicle initiation or tillering stages for improvement in growth and yield of rice with and without AMF inoculation.

## Material and methods

### Experimental site and design

A pot study was conducted in the research area of the Department of Soil Science (71.43^o^ E, 30.2^o^ N and 122 meters above sea level), Bahauddin Zakariya University Multan.

### Treatments

There were four Zn application treatments i.e., control (foliar application of tap water (TW)), 0.5% Zn foliar spray at tillering stage (0.5ZnT), 0.5% Zn foliar spray at panicle stage (0.5ZnP) and 0.5% Zn foliar spray at panicle and tillering stages (0.5ZnP+T). While two levels of AMF were used in the study including No AMF (no AMF inoculated) and AMF. The treatment plan includes TW+AMF, 0.5ZnT+AMF, 0.5ZnP+AMF, 0.5ZnP+T+AMF, TW, 0.5ZnT, 0.5ZnP and 0.5ZnP+T. The experimental treatments were laid out in a completely randomized design (CRD) under the factorial arrangement, and each treatment was replicated three times.

### Pots preparation and soil characterization

Clay pots were utilized for the experiment having 60 cm depth and 45 cm diameter. The soil was sampled from the experimental area. After sieving from a 2mm sieve, 8 kg soil was filled in each pot. A composite sample was also taken for the characterization of soil attributes. The texture was analyzed through the determination of sand, silt and clay; the textural triangle of USDA was utilized for computation of soil texture [21]. For analysis of pH, soil and deionized water paste was made by missing in 1:1 ratio. After that pH of saturated paste was computed using a pre-calibrated pH meter [22]. For assessment of soil EC, 1:10 ratio soil and distilled water mixture were prepared. Extraction was done and then EC of the extract was noted on pre-calibrated (1/100N KCl) EC meter [23]. Ferrous ammonium sulphate and potassium dichromate were utilized for the analysis of soil organic matter [24]. The soil sample was digested at 380°C on the hot plate for analysis of total nitrogen by Kjeldhal’s distillation apparatus [25]. For assessment of available phosphorus, Olsen extraction (sodium bicarbonate) was done. Final P was examined on a spectrophotometer at 880nm wavelength [26]. Potassium was examined in the ammonium acetate soil extract on a flame photometer by following the protocol of [27]. For analysis of Zn in soil, DTPA extract was done. The final analysis was performed on atomic absorption spectrophotometer (AAS) [28]. The pre-experimental soil attributes are provided in Table 1.

**Table 1:** Physico-chemical properties of experimental soil.

Soil			Water		
Attributes	Units	Values	Attributes	Units	Values
Sand	%	55	EC	μS cm^-1^	360
Silt		15	Carbonates	meq./L	0.00
Clay		30	Bicarbonates		1.02
Texture	Sandy Clay Loam				
pH*s*	-	8.23	Chlorides		0.10
EC*e*	dS/m	4.76	Ca+Mg		5.61
Organic matter	%	0.45	Soluble Zinc	mg kg^-1^	0.10
Total Nitrogen	%	0.023	pH	-	6.89
Available phosphorus	mg kg^-1^	6.55			
Extractable potassium		157			
Extractable zinc		11.23			

### Seed purchasing and nursery development

Seed of SUPER BASMATI rice variety was purchased from the certified seed dealer for the plantation of rice nursery. After 25 days of germination, seedlings were transplanted in the pots.

### AMF inoculation

For AMF inoculation, 10 kg soil was inoculated with 2.5 g mycorrhizal inoculum Clonex® (Root Maximizer; 5711 Enterprise Drive, Lansing, MI, USA). The commercial product had 158 propagule gram^-1^ with Glomus species, as a major ingredient of the product. At the time of transplantation, AMF inoculation was again applied to the seedling in treatment with AMF application for maximum colonization [1, 10].

### Zinc foliar spray

For the foliar application of Zn, salt of ZnSO_4_ was utilized. Each treatment at respective application stages i.e., panicle and tillering received 0.5% Zn solution. The solution of Zn was made in tap water. The characteristics of tap water are also provided in Table 1. For control, only tap water was sprayed during treatment application at panicle and tillering stages.

### Fertilizer application and irrigation

Recommended macronutrients including N, P and K as urea, sulfate of potash (SOP) and diammonium phosphate (DAP) were applied at the rate of 0.84, 0.54 and 0.36g. The N fertilization was done in three splits; half of the total recommended N was added at the time of sowing, while the remaining half was applied in 2 splits i.e., tillering and spike initiation stages [31]. In each pot, 100% FC of water was maintained throughout the experiment [32].

### Gas exchange attributes

Gas exchange attributes were determined by utilizing IRGA [CI-340 Photosynthesis system, CID, Inc. USA] as described by Danish and Zafar-ul-Hye [29] at 45 days after germination. The readings were collected in 45 days old rice plants on a sunny day with an intensity of light saturation between 10:33 and 11:10 AM.

### Chlorophyll contents and electrolyte leakage

For chlorophyll contents assessment, Arnon [30] method was followed. Electrolyte leakage was assessed according to the methodology of [31]. Final calculations were made by using the following equation for electrolyte leakage

$$EL\;(\%)=\frac{EC1}{EC2}\times 100$$ (1)

### Data collection

Plants were harvested at the time of maturity. Morphological attributes i.e., number of spikes, plant height, 1000 grains weight and spike length were recorded soon after harvesting of the crop. Grains and straw yield were noted via manual separation of grains and straw. After that top weight balance was use for the assessment of grains and straw yield.

### Grains nutrients concentration

Nitrogen in grains was computed by digestion of sample at 400°C with H_2_SO_4_. After digestion distillation was done on Kjeldhal’s distillation apparatus [32]. For phosphorus (P) and potassium (K) in grains and straw, digestion was done with di-acid mixture (HNO_3_:HClO_4_ = 2:1) [33]. Yellow colour method was used for the final examination of P on the spectrophotometer [34] while a flamephotometer and atomic absorption spectrophotometer were used for K and Zn determination respectively [35, 36].

### Statistical analysis

The standard statistical procedure was followed for statistical analysis of data [37]. Data collected were statistically analyzed using two-way factorial ANOVA. While comparison of each treatment was made by applying the Fisher LSD test (p≤0.05). Pearson correlation was also computed, and probability graphs were made by using OriginPro 2021 [38].

## Results

Effects of treatments were significant on AMF colonization with roots, plant height, spike length and number of spikes. Results showed that 0.5ZnT+P with AMF remained significantly better compared to all other treatments for the improvement in AMF root colonization. Treatment 0.5ZnT and 0.5ZnP also differed significantly over control (TW+AMF) for AMF colonization with roots. No significant change in AMF colonization with roots was observed where TW and 0.5ZnT were apploed as treatments. However, 0.5 ZnP and 0.5 ZnT+P performed significantly better than the control (TW) for enhancement in AMF colonization with roots compared to TW (Fig 1A). For enhancement in plant height, 0.5ZnT+P and 0.5ZnP with AMF remained significantly better than TW. A significant improvement in plant height was also observed in 0.5ZnT with AMF than TW. It was observed that 0.5ZnT+P, 0.5ZnP and 0.5ZnT differed significantly over TW without AMF for enhancement in plant height (Fig 1B). In the case of spike length and number of spikes, 0.5ZnT+P, 0.5ZnP and 0.5ZnT caused a significant increase compared to TW with AMF. Treatments 0.5ZnT+P and 0.5ZnP differed significantly for spike length (Fig 1C) and number of spikes (Fig 1D) over TW without AMF. However, no significant change in spike length and number of spikes was noted where 0.5ZnT was applied than TW without AMF.

**Fig 1:** Effect of zinc foliar application at tillering and panicle stages with and without AMF inoculation on AMF colonization with roots (A), plant height (B), spike length (C) and number of spikes (D) of rice. Bars are means of three replicates ± SE. Variable letters on bars indicate significant difference at p ≤ 0.05 according to LSD test. TW = tap water (control); T = tillering stage; P = panicle stage; Zn = zinc.

The influences of treatments were significant on 1000 grains weight, total chlorophyll and electrolyte leakage. Application of 0.5ZnT+P and 0.5ZnP with and without AMF was significantly different than TW for the enhancement in 1000 grains weight. No significant change was noted in 0.5ZnT with and without AMF for 1000 grains weight than TW (Fig 2A). Treatments 0.5ZnT+P, 0.5ZnP and 0.5ZnT remained significantly better for total chlorophyll compared to TW with and without AMF. Treatments 0.5ZnP and 0.5ZnT remained statistically alike to each other for total chlorophyll in the absence and presence of AMF (Fig 2B). It was noted that 0.5ZnT did not differ significantly for a decrease in electrolyte leakage compared to TW when applied with AMF. However, 0.5ZnT+P and 0.5ZnP with AMF caused a significant decrease in electrolyte leakage over TW. A significant decrease in electrolyte leakage was noted where 0.5ZnT+P, 0.5ZnP and 0.5ZnT without AMF were applied compared to TW (Fig 2C).

**Fig 2:** Effect of zinc foliar application at tillering and panicle stages with and without AMF inoculation on 1000 grains weight (A), total chlorophyll (B) and electrolyte leakage (C) in rice leaves. Bars are means of three replicates ± SE. Variable letters on bars indicate significant difference at p ≤ 0.05 according to LSD test. TW = tap water (control); T = tillering stage; P = panicle stage; Zn = zinc.

The addition of treatments caused a significant change in gas exchange attributes i.e., photosynthetic rate, transpiration rate and stomatal conductance. Application of 0.5ZnT+P and 0.5ZnP with and without AMF remained significantly different than TW for the photosynthetic rate. Treatment 0.5ZnT did not differ significantly for photosynthetic rate compared to TW. Results also showed that 0.5ZnT+P, 0.5ZnP and 0.5ZnT without AMF were significantly better over TW for photosynthetic rate (Fig 3A). A significant change was noted in transpiration rate where 0.5ZnT+P, 0.5ZnP and 0.5ZnT with AMF were applied compared to TW. Compared to TW, 0.5ZnT+P and 0.5ZnP were significantly different but 0.5ZnT showed the non-significant change in transpiration rate without AMF (Fig 3B). It was noted that 0.5ZnT remained non-significant for stomatal conductance than TW when applied with AMF. However, 0.5ZnT+P and 0.5ZnP with AMF differed significantly better over TW for enhancement in stomatal conductance. A significant increase in stomatal conductance was observed in 0.5ZnT+P, 0.5ZnP and 0.5ZnT without AMF over TW (Fig 3C).

**Fig 3:** Effect of zinc foliar application at tillering and panicle stages with and without AMF inoculation on photosynthetic rate (A), transpiration rate (B) and stomatal conductance (C) in rice leaves. Bars are means of 3 replicas ± SE. Variable letters on bars indicate significant difference at p ≤ 0.05 according to LSD test. TW = tap water (control); T = tillering stage; P = panicle stage; Zn = zinc.

It was noted that grains and straw yields were also significantly changed by the addition of treatments. A significant improvement in grains (Fig 4A) and straw yield (Fig 4B) was noted in 0.5ZnT+P, 0.5ZnP and 0.5ZnT with and without AMF over TW. On average, application of treatments with AMF performed significantly better than without AMF for grains and straw yields.

**Fig 4:** Effect of zinc foliar application at tillering and panicle stages with and without AMF inoculation on rice grains yield (A) and straw yield (B). Bars are means of three replicates ± SE. Variable letters on bars indicate significant difference at p ≤ 0.05 according to LSD test. TW = tap water (control); T = tillering stage; P = panicle stage; Zn = zinc.

Application of treatments also caused a significant change in grains N, P, K and Zn accumulation. The addition of 0.5ZnT+P and 0.5ZnP with and without AMF performed significantly better than TW for enhancement in grains N. Treatment 0.5ZnT with and without did not cause any significant change in grains N over TW. For grains P, 0.5ZnT+P cause a significant increase compared to TW (Table 2). Treatments 0.5ZnP and 0.5ZnT were statistically alike with TW in the presence and absence of AMF for grains P. In the case of grains K and Zn, 0.5ZnT+P, 0.5ZnP and 0.5ZnT with and without AMF caused a significant increase over TW (Table 1). Compared to TW, the maximum increase in N (14.5 and 25.7%), P (42.1 and 33.3%), K (22.2 and 30.0%) and Zn (19.3 and 27.8%) was noted in ZnT+P with and without AMF respectively.

**Table 2:** Effect of zinc foliar application at tillering and panicle stages with and without AMF inoculation on rice grains nitrogen, phosphorus, potassium and zinc.

Inoculation	Zinc	Grains Nitrogen (%)			Grains Phosphorus (%)		
		Mean	SE	Labelling	Mean	SE	Labelling
AMF	TW	11.58	0.31	d	0.19	0.002	bcd
AMF	0.5Zn T	12.11	0.06	bcd	0.23	0.015	ab
AMF	0.5Zn P	12.42	0.21	bc	0.24	0.007	ab
AMF	0.5Zn T+P	13.26	0.16	a	0.27	0.036	a
No AMF	TW	10.14	0.04	e	0.15	0.003	d
No AMF	0.5Zn T	10.51	0.29	e	0.17	0.003	cd
No AMF	0.5Zn P	11.81	0.41	cd	0.18	0.003	cd
No AMF	0.5Zn T+P	12.75	0.16	ab	0.20	0.003	bc
Inoculation	Zinc	Grains Potassium (%)			Grains Zinc (μg g^-1^)		
		Mean	SE	Labelling	Mean	SE	Labelling
AMF	TW	0.21	0.003	d	26.18	0.47	c
AMF	0.5Zn T	0.23	0.003	c	28.18	0.10	b
AMF	0.5Zn P	0.26	0.003	ab	28.72	0.36	b
AMF	0.5Zn T+P	0.27	0.003	a	31.22	0.63	a
No AMF	TW	0.20	0.003	e	18.67	0.33	g
No AMF	0.5Zn T	0.23	0.006	c	20.67	0.33	f
No AMF	0.5Zn P	0.25	0.003	b	22.00	0.58	e
No AMF	0.5Zn T+P	0.26	0.003	ab	23.67	0.33	d

Values are means of 3 replicas ± SE. Variable letters showed significant difference at p ≤ 0.05 compared by using Fisher LSD test. TW = tap water (control); T = tillering stage; P = panicle stage; Zn = zinc.

Pearson correlation showed that AMF root colonization was significantly and positively correlated with plant height, spike length, number of spikes, 1000 grains weight, total chlorophyll, photosynthetic rate, transpiration rate, stomatal conductance, straw yield, grains N, P and Zn concentration. It was also noted that only electrolyte leakage was significant negatively correlated with AMF root colonization and grains Zn concentration. Grains yield was significantly positive in correlation with photosynthetic rate, spikes length, N, P, K concentration in grains and stomatal conductance (Fig 5).

**Fig 5:** Pearson correlation for studied rice growth attributes affected zinc application at different growth stages.

## Discussion

Results of the current study confirmed that application of 0.5% foliar Zn at tillering+panicle stages with AMF significantly enhanced plant height, spike length, number of spikes and 1000 grains weight. The development of symbiosis between plants roots and fungal hyphae significantly enhanced the expansion of roots. Better elongation in roots resulted in optimum uptake of water and nutrients which ultimately improved plant growth [39, 40]. Better root colonization of plants with AMF also positively affected pollen delivery, pollen germination, pollen tube growth, fertilization and germination of seeds [41]. A significant increase in mineral nutrient uptake due to inoculation of AMF in plants is also a key feature that caused improvement in the yield of crops [42]. A similar trend of nutrient improvement was also recorded in current. It was observed that grains N, P, K and Zn concentration was significantly high where 0.5ZnT+P with AMF was applied over control. The improvement in grain’s nutrients was due to mutual positive effects of ZnT+P and AMF. Inoculation of AMF in soil decrease N losses as leaching due to promotion of aggregates formation as a result of organic secretions. Better soil aggregates also facilitate the penetration of air thus minimizing the effects of denitrification N losses. On the other hand, a strong correlation between N uptake and chlorophyll contents regulates the rubisco activity during photosynthesis. This improvement in photosynthesis is also dependent on CO_2_ assimilation rate through optimization of stomatal conductance in the plants [43, 44]. Application of 0.5ZnT+P with AMF caused significant improvement in chlorophyll contents and gas exchange attributes i.e., photosynthetic rate and stomatal conductance. The improvement was more prominent in the presence of AMF compared to No AMF. Furthermore, deficiency of Zn also decreases K ions concentration in the guard cells. Such increase in K ions efflux compared to influx caused damage to cell membrane under deficient Zn conditions [45]. However, the role of Zn at tillering+panicle was also significant in the enhancement of chlorophyll contents, photosynthetic rate and stomatal conductance. Balance uptake of Zn in plants improves membrane integrity. This improvement in membrane integrity regulates the stomatal conductance in plants [45]. It has also been observed that less Zn uptake minimize the activity of carbonic anhydrase. The reduction in this activity adversely affects the photosynthesis in plants through disturbance in PS-II and disintegration of Rubisco structure [46, 47]. In the current study, it was noted that AMF also facilitates the better uptake of Zn in grains. This improvement was due to tradeoff mechanism of AMF regarding plant nutrients and Zn uptake. According to this mechanism, AMF inoculation increases the uptake of Zn when plants are cultivated in Zn deficient soils. On the other hand, higher Zn concentration can also cause toxicity in the plants. Inoculated AMF in the current situation played an imperative role in decreasing Zn uptake to provide some relaxation in toxicity for crops [1, 10]. A significant decrease in electrolyte leakage of rice leaves in the current study also validated the above mechanism of balance Zn and other nutrients uptake. As plants were cultivated in Zn deficient soil, the higher electrolyte leakage was associated with the deficiency of Zn. Similarly, the grains Zn was also poor compared to 0.5ZnT+P in the presence and absence of AMF validated the fact of Zn stress in rice plants. According to Matile et al. [48], chlorophyllase activation in the chloroplast played notorious role in the destruction of chlorophyll after direst contact of stress ethylene with cell membrane. Under stress conditions, this stress ethylene become accumulated and degrade the lipid membrane due to which membranes loss their integrity [48]. This might be associated with low chlorophyll contents in control and high electrolyte leakage.

## Conclusions

Foliar application of Zn at tillering and panicle initiation stages improved the growth and yield of rice than control. However, such effects were provoked with AMF inoculation. Sole application of Zn at panicle initiation stage was more effective than its application at tillering for improvement in 1000 grains weight, and grains nutrient accumulation. In crux, foliar Zn application at tillering+panicle stages with AMF inoculation is better to approach compared to sole application for significant improvement in rice growth and yield. It is suggested to grower to inoculate AMF and apply 0.5%Zn foliar at tillering+panicle stages for better rice crop growth. However, more investigations are suggested on different cereal crops under the agroclimatic zone to declare foliar 0.5%Zn at tillering+panicle as the best treatment.
